# Oral Cancer Incidence, Mortality, and Mortality-to-Incidence Ratio Are Associated with Human Development Index in China, 1990–2019

**DOI:** 10.1155/2022/6457840

**Published:** 2022-06-28

**Authors:** Long Xie, Zheng-Jun Shang

**Affiliations:** ^1^The State Key Laboratory Breeding Base of Basic Science of Stomatology (Hubei-MOST) & Key Laboratory of Oral Biomedicine Ministry of Education, School & Hospital of Stomatology, Wuhan University, Wuhan, China; ^2^Department of Oral and Maxillofacial-Head and Neck Oncology, School and Hospital of Stomatology, Wuhan University, 237 Luoyu Road, Wuhan 430079, China

## Abstract

The burden of oral cancer (OC) is closely related to economic development. We aimed to evaluate the burden of OC at different stages of economic development in China in terms of incidence, mortality, and mortality-to-incidence ratio (MIR) from 1990 to 2019. Data on cancer in China from 1990 to 2019 were obtained from the Global Burden of Disease 2019. Based on human development index (HDI), Chinese economic development was divided into three stages: low, medium, and high HDI stages. Mann–Whitney *U*-test was used to evaluate the differences in age-standardised incidence rates (ASIR), age-standardised mortality rates (ASMR), and MIR at various stages of HDI. Correlation and regression tests were conducted to examine the association amongst ASIR, ASMR, MIR, and HDI in OC. The estimated annual percentage changes (EAPCs) were calculated to assess the trend of ASIR, ASMR, and MIR. Significant differences were observed in terms of ASIR, ASMR, and MIR between groups (*P* < 0.001). The values of both sexes in the low HDI stage were lower than those of the medium and high HDI stages, except for MIR, in which the low HDI stage was the highest (*P* < 0.05). ASIR and ASMR of OC in males at the medium HDI stage showed the fastest growth rate with EAPC values of 5.64 (95% confidence interval, 95% CI, 5.20 to 6.08) and 4.42 (95% CI, 4.01 to 4.82), respectively. A strong positive correlation exists between HDI and ASIR (*r* = 0.96) and ASMR (*r* = 0.91) in both sexes from 1990 to 2019. During the high HDI stage, the ASIR and ASMR of OC were at a high level, but the ASIR halted the uptrend trend and ASMR showed a decreasing trend. Therefore, the HDI index has been positively correlated with the ASIR and ASMR of OC in China in the past 30 years, but this relationship may not be sustained as the economy develops. The health department should continue to allocate additional resources for the prevention and treatment of OC.

## 1. Introduction

Oral cancer ranks sixth most prevalent type of cancer worldwide due to its rapid increase every year [1]. Over 450,000 patients worldwide are diagnosed with OC annually, and it has a five-year survival rate of under 50% [2, 3]. The incidence of total OC increased slightly from 1990 to 2017, whilst death rate remained stable [4]. However, these characteristics vary amongst countries; OC incidence and death rates in China increased from 2005 to 2013, and crude incidence rates will increase from 2.26 to 3.21 per 100,000 over the next 20 years [5]. Globocan 2020 estimates indicate that the age-standardised rates of OC morbidity and mortality ranked 20th and 22nd amongst all cancers in China in 2020 [6].

The causes of OC are complex. Approximately 90% of head and neck cancers are linked to smoking, drinking, and poor diet [7]. A meta-analysis has suggested that smokers are five times more likely to develop OC than nonsmokers [8]. Although drinking alcohol increases the risk of oral cancer by 1.56 times, higher rates of advanced oral cancer are associated with combined use of tobacco and alcohol [9, 10]. Other studies have shown that betel nut and HPV virus infections are also closely related to oral cancer [9, 11].

With the development of the economy, people's ability to consume will increase (including the consumption of tobacco and alcohol). Cancer spectrum in China also presents new changes, from infectious diseases to noncommunicable diseases (including OC) [12]. The decline in fertility, acceleration of urbanisation, and increase in life expectancy had led to major changes in the demographic structure, leading to a corresponding increase in the burden of noncommunicable diseases, including cancer [13]. The incidence of cancer is also closely related to national economic development. Human development index (HDI) is an independent predictor of tumour burden. For example, HDI index is positively correlated with age-standardised incidence rates (ASIR) and age-standardised mortality rates (ASMR) of lung cancer [14]. High and medium HDI countries had seen a disproportionate increase in the disease burden of OC [15]. Whether the HDI index is correlated with the incidence and mortality of OC in developing country like China is worthy of investigation.

Reports on the relationship between HDI and OC at different stages of economic development in China are scarce. In recent years, the number of cases of OC has been increasing, and the burden of OC has become heavier, bringing a heavy burden to the country and the family with OC patients. It is urgent to analyse the correlation between HDI index and the burden of OC and make corresponding adjustments to health policies in the future. Hence, the current study aims to analyse the effect of HDI on ASIR, ASMR, and mortality-to-incidence ratio (MIR) of OC between 1990 and 2019 in China.

## 2. Materials and Methods

### 2.1. Date Source

Data on the burden imposed by OC in China were obtained from the Global Burden of Disease (GBD) 2019 study (http://ghdx.healthdata.org/gbd-results-tool) for 1990−2019 in China. MIR was calculated by dividing ASMR by ASIR.

Chinese HDI data for 1990−2019 were obtained from the United Nations Development Programme (UNDP) database. HDI, which includes life expectancy at birth, average and expected years of education, and per capita national income, involves three parameters. The values ranged from 0 to 1. HDI has four categories: very high (HDI>0.800), high (0.700 < HDI <0.799), medium (0.550 < HDI<0.699), and low (HDI<0.550). Given that the HDI data of China in 2019 did not reach 0.8, its economic development from 1990 to 2019 was divided into three stages according to HDI data. The periods 1990–1996, 1997–2010m and 2011–2019 refer to low, medium, and high HDI stages.

The following country-specific healthcare parameters were derived from the National Bureau of Statistics database of China (https://data.stats.gov.cn/index.htm): health expenditure as %age of GDP (CHE) in calendar years, out-of-pocket expenditure as %age of total health expenditure (OOP), number of certified doctors (NCD) per 10,000 population and per capita health expenditure (HE), and cigarette, liquor, and beer production.

### 2.2. Statistical Analyses

The statistical analysis was implemented using the R programming language (Version 3.6.2). More exactly, Mann–Whitney *U*-test was used to evaluate the differences in ASIR, ASMR, and MIR at various stages of HDI, and the relationship of HDI to ASIR, ASMR, and MIR using univariate linear regression. A significant difference was considered regarded when *P* < 0.05.

Estimated annual percentage changes (EAPCs) were used to describe ASR trend within a specified time interval [16]. The natural logarithm of ASR has a linear relationship with time, in which *Y* = *α* + *βX* + *ε*, where *Y* refers to ln (ASR), *X* stands for the calendar year, and *ε* is an error term. According to this formula, *β* indicates positive or negative trends in ASR. EAPC is calculated as follows: EAPC = 100 × (exp (*β*)–1). The calculation formula of EAPC and its 95% confidence interval were obtained from the linear model. When the lower limits of confidence interval and EAPC are positive, ASR has an upward trend. Conversely, when the upper limits of the confidence interval and EAPC are negative, ASR has a descending trend.

## 3. Results

Table 1 shows the number of cases, deaths, morbidity, mortality, ASIR, ASMR, and MIR of OC in terms of sex and HDI stage from 1990 to 2019.

Table 2 shows that the number of cases and deaths from OC increased from 1990 to 2019, with the highest increase occurring at the medium HDI stage. The most significant increase was that the number of cases and deaths of male patients increased by 128.86% and 111.75%, respectively, at the medium stage. At the low and medium HDI stages, ASIR of males showed an upward trend, with EAPC values of 3.75 (95% CI, 3.39, 4.11) and 5.64 (95% CI, 5.20, 6.08), respectively. For the same periods, ASMR showed an upward trend, with EAPC values of 2.79 (95% CI, 2.48, 3.11) and 4.42 (95% CI, 4.01, 4.82), respectively. Although the number of cases and deaths from OC increased in females, the incidence of OC decreased at the low HDI stage, with an EAPC of −0.40 (95% CI, −0.79, −0.01). At the high HDI stage, ASIR maintained a stable trend, while ASMR showed a decreased trend. At all stages, MIR showed a downward trend, and the difference was statistically significant.

Figure 1 shows the comparison of the three HDI stages in terms of both sexes' morbidity, mortality, ASIR, ASMR, and MIR. The Mann–Whitney *U*-test showed significant differences in terms of incidence, mortality, ASIR, ASMR, and MIR between groups (*P* < 0.001). The Mann–Whitney *U* test revealed that in all indicators, values of the low HDI stage were lower than those of the medium and high HDI groups (*P* < 0.05), except for MIR, in which the low HDI stage was the highest (*P* < 0.001).

Figure 2 shows the annual output of tobacco, liquor, and beer at the medium HDI stage is lower than that at the high HDI stage (*P* < 0.001).

Figure 3 presents the scatterplots of HDI versus ASIR, ASMR, and MIR. It is shown that HDI is positively correlated with ASIR and ASMR and negatively correlated with MIR when both sexes are considered together (Figure 3(a)–(c)). The patterns of the relationships stay very similar when the male is exclusively considered. Moreover, the slopes are quite large for those positive correlations (9.24 for ASIR, and 4.28 for ASMR) and small for the negative correlation (-0.653 for MIR). In contrast, the female data show all negative correlations and mild slopes (-0.125 for ASIR, -0.721 for ASMR, -0.571 for MIR).

Figure 4 lists the correlations amongst HDI, ASIR, ASMR, and MIR whether male and female data are considered simultaneously or separately. The red colour indicates a negative correlation while the blue colour indicates a positive correlation. The size of the circle indicates the absolute value of the correlations. It is found that the correlations amongst HDI, ASIR, ASMR, and MIR for male or for both genders together are close to +1 or -1, indicating a strong positive (e.g., HDI and ASIR, HDI, and ASMR) or negative correlation (e.g., HDI and MIR). The correlations amongst HDI, ASIR, ASMR, and MIR for females sometimes are far from +1 or -1 (e.g., -0.42 for HDI and ASIR).

Figure 5 shows that MIR is related to country-specific healthcare parameters. MIR was negatively correlated with CHE (*r* = −0.916, *P* < 0.001), HE (*r* = −0.916, *P* < 0.001) and NCD (*r* = −0.775, *P* < 0.001) and negatively positively with OOP (*r* = 0.633, *P* < 0.001). It should be noted that the relationship between OOP and MIR is twofold: positive correlation when MIR<0.62 and negative correlation otherwise. The reason is that in 2002, the Chinese government began to solve the economic burden of catastrophic diseases in rural residents through the new rural cooperative medical system, and the proportion of reimbursement gradually increased since 2002 [17].

## 4. Discussion

OC is a major cause of cancer morbidity and mortality in China, and crude incidence rates will increase over the next 20 years [5]. In this research, Chinese economic development from 1990 to 2019 was divided into three stages according to HDI. Thereafter, the trends of ASIR, ASMR, and MIR in three stages and the correlation between HDI and ASIR, ASMR, and MIR of OC based on GBD data were analysed. Lastly, the correlation between MIR and country-specific healthcare parameters was determined.

The results showed that the incidence and mortality of OC vary from one stage to another and were highest at the high HDI stage. The findings of some studies were consistent with our results. Brazil and Cuba, which had high HDI and high tobacco and alcohol consumption, have high rates of OC morbidity and mortality [18, 19]. In our country, the annual output of tobacco, liquor, and beer at the high HDI stage was higher than that at the medium HDI stage. That is, the development of the economy resulted in a substantial increase in the domestic consumption of tobacco and alcohol (Figure 2). Countries with high HDI also have more elderly people than countries with low HDI [20]. On the one hand, long-term exposure of the elderly to various complex environments and risk behaviour factors leads to increased incidence of cancer [21]. On the other hand, the prevalence of systemic comorbidities in patients with OC increased from 0.820% (2003) to 32.302% (2017) with the development of the economy and society, causing an increased risk of death [22]. The highest morbidity and mortality of OC at the high HDI stage may be attributed to the accurate registration system for cancer [23].

The present study found that at the medium HDI stage, the proportion of morbidity and mortality increased the most, whilst at the low and medium HDI stages, morbidity and mortality in males showed an upward trend. With the emergence of industrialisation, emissions of fine particulate matter (PM) had increased, and exposure to high concentrations of PM2.5 had increased the risk of OC [24, 25]. For example, the annual average concentration of PM2.5 in Beijing from 2001 to 2003 was even as high as 154.3 *μ*g/m^3^ [26]. Morbidity and mortality rates from OC were higher in men than in women because of tumour-related risk factors, such as smoking and alcohol consumption and diagnosis of late clinical stage [9, 27]. The decreasing incidence of OC in females at the low HDI stage may be attributed to the fact that women in China traditionally avoid smoking and alcohol. At the high HDI stage, ASIR maintained a stable trend with EAPC value of -0.21(95% CI, -0.49, 0.06), and ASMR maintained a down trend with EAPC value of -1.33(95% CI, -1.75, -0.91). At the high HDI stage, tobacco control actions in China were strengthened, smoking rates were reduced, and cessation rates increased, thereby curbing and levelling off the increasing incidence and mortality of OC [28]. Furthermore, with economic development, the state increased funds to the treatment of OC, reduced the burden on patients, and improved the survival rate. With the vigorous development of oral medicine, the ability to diagnose and treat OC has been further improved [29]. The Chinese government has been investing heavily to combat pollution. Over $277 billion were pledged by the Academy for Environmental Planning in 2013. Between 2013 and 2017, the levels of PM2.5 were reduced by 33 per cent in at least 74 cities. The following year, it fell by a further 10 per cent. During August 2019, Beijing experienced the lowest PM2.5 reading since records began. It stood at just 23 *μ*g/m^3^ [30]. Effective air therapy measures also help reduce the incidence and mortality of OC in China.

HDI was positively correlated with ASIR and ASMR in both sexes. With the development of the economy, the incidence and mortality of OC increased. This correlation was consistent with epidemiologic transition theory, which states that as different stages of socioeconomic development mature, communicable diseases gradually give way to the doctrine of noncommunicable diseases [31]. As the country transitions to a high level of human development, the behaviour of the general population has leaned to traditional lifestyles and built environments prevailing in high-income and Westernised societies. HDI is positively associated with percentage of overweight adults with OC. A sedentary lifestyle, increasing prevalence of obesity, changes in eating habits and reproductive patterns, and other Western lifestyle choices increased OC mortality rates [32].

It should be noted that in Figures 3(a), 3(b), 3(d), and 3(e), ASMR showed a downward trend and ASIR showed a stable trend at the high HDI stage. Economic development was significantly associated with OC in each country. Incidence of OC was closely related to GDP per capita, with a negative correlation in countries with GDP per capita (at purchasing power parity) above US$10,000 and a positive correlation in countries with GDP per capita below US$10,000 (at purchasing power parity) [33]. The World Bank database indicated that at the low and medium HDI stages in China, GDP per capita was under US$10,000. By contrast, GDP per capita started to reach or exceed US$10,000 (at purchasing power parity) at the high HDI stage. These findings can explain the decreasing trend of ASMR and the halted uptrend of ASIR in the high HDI stage of OC, as shown in Figures 3(a), 3(b), 3(d), and 3(e). From 2005 to 2014, Brazil was at a high HDI stage, and ASMR of OC was negatively correlated with HDI [32]. This finding may be associated with increased attention to oral health at the high HDI stage and with the reduction of advanced OC through early screening. This result can explain the decreasing trend of ASMR of male OC at the high HDI stage, as shown in Figure 3(e). ASIR and ASMR of OC in women were slightly inversely associated with HDI (Figures 3(g) and 3(h) and Figure 4). The possible reasons were increased awareness of oral healthcare, early screening, reduced consumption of tobacco and alcohol, and advancements in medical technology.

The present study showed that MIR has an inverse relationship with HDI (Figures 3(c), 3(f), and 3(i)). MIR was an indicator of the effectiveness of health systems and recommended as an indirect criterion to measure actual biological differences in disease phenotypes or health system-related features, such as screening, diagnostic methods, treatment, and follow-up [34]. Low CHE, HE, and NCD and high OOP indicate the weakness of the healthcare system (Figure 5). At the low HDI phase, patients were at a relative disadvantage period because of late diagnosis, unavailability of treatment options, and high treatment costs, most of which were paid out of their pocket. The correlation between MIR and HDI in OC can also be verified in other tumours. Hu showed countries with low HDI have the highest MIR of female breast cancer [35]. HDI exhibited a negative significant relationship with MIR at the tumour site of lungs, liver, and colorectal [36–38]. In China, differences in MIR may be attributed to unequal access to health services or different national investments in health resources annually. Meanwhile, differences in the quality of mortality and morbidity data at each stage were linked to differences in MIR.

Some limitations of this study are as follows. Firstly, GBD obtained data from various sources, such as vital registries, cancer registries, and verbal autopsies through multiple modelling steps detailed elsewhere [39, 40]. Incidence and death rates of OC from the GBD database may differ from the actual data. Secondly, the GBD database provided 30 years of OC data in China. According to HDI, the corresponding data of 30 years from 1990 to 2019 were divided into three groups. Data in each group were not equal, thereby affecting the analysis of the results. Lastly, the results of this study cannot be generalised to other countries considering the special attributes of China (e.g., world largest population).

Our study is the first to analyse the association of China's economic index HDI with oral cancer disease burden. During the high HDI stage, the ASIR and ASMR of OC were at a high level, but the ASIR halted the uptrend trend and ASMR showed a decreasing trend. Our study found the HDI index has been positively correlated with the ASIR and ASMR of OC in China in the past 30 years, but this relationship may not be sustained as the economy develops. The health department should continue to devote additional resources for the prevention and treatment of OC.

## Figures and Tables

**Figure 1:** The comparison of the three HDI stages in terms of ASIR, ASMR, and MIR. The Mann–Whitney *U*-test showed significant differences of ASIR, ASMR, and MIR between groups (*P* < 0.001). ∗P < 0.05 Mann–Whitney *U*-test between groups; ∗∗P < 0.01 Mann–Whitney *U*-test between groups; ∗∗∗P < 0.001 Mann–Whitney *U*-test between groups.

**Figure 2:** Production of tobacco, liquor, and beer at medium and high HDI stages. All the data are derived from the National Bureau of Statistics database of China (https://data.stats.gov.cn/index.htm).

**Figure 3:** The scatterplots of HDI versus ASIR, ASMR, and MIR by gender. (a, d, g) represent HDI vs ASIR by gender; (b, e, h) represent HDI vs ASMR by gender; (c, f, i) represent HDI vs MIR by gender.

**Figure 4:** Correlation matrix map of the four variables: HDI, ASIR, ASMR, and MIR by gender.

**Figure 5:** Correlation between MIR and country-specific healthcare parameters. (a) MIR vs CHE, (b) MIR vs HE, (c) MIR vs NCD, (d) MIR vs OOP. MIR: mortality-to-incidence ratio; CHE: health expenditure as %age of GDP; HE: per capita health expenditure (Yuan); NCD: number of certified doctors per 10:000 population; OOP: out-of-pocket expenditure as %age of total health expenditure. The corresponding data of MIR, CHE, HE, UHC, and OOP are from 1990 to 2019. All the data are derived from the National Bureau of Statistics database of China (https://data.stats.gov.cn/index.htm).

**Table 1:** Number, crude, and standardised incidence rates, mortality, and MIR from oral cancer in China from 1990 to 2019.

Time	Gender	ASIR	ASMR	All age death numbers	All age incidence number	All age incidence rate	All age death rate	Mortality-to-incidence ratio
Low HDI	Both sex							
1990		1.40	0.92	7403	12390	1.05	0.63	0.66
1991		1.41	0.92	7599	12807	1.07	0.63	0.65
1992		1.40	0.91	7716	13034	1.07	0.64	0.65
1993		1.41	0.91	7898	13427	1.10	0.64	0.65
1994		1.40	0.91	8056	13748	1.11	0.65	0.65
1995		1.40	0.90	8193	14078	1.13	0.66	0.64
1996		1.40	0.89	8329	14461	1.15	0.66	0.64
Medium HDI								
1997		1.38	0.87	8418	14733	1.16	0.66	0.63
1998		1.38	0.87	8604	15168	1.18	0.67	0.62
1999		1.40	0.87	8915	15780	1.22	0.69	0.62
2000		1.44	0.89	9420	16684	1.28	0.72	0.62
2001		1.48	0.91	9897	17566	1.34	0.76	0.62
2002		1.53	0.93	10492	18650	1.42	0.80	0.61
2003		1.61	0.97	11290	20145	1.52	0.85	0.61
2004		1.69	1.01	12174	21884	1.65	0.92	0.60
2005		1.75	1.04	12881	23293	1.74	0.96	0.59
2006		1.80	1.06	13518	24678	1.84	1.01	0.59
2007		1.87	1.08	14302	26391	1.96	1.06	0.58
2008		1.96	1.12	15357	28553	2.11	1.13	0.57
2009		2.07	1.17	16548	31012	2.28	1.22	0.57
2010		2.19	1.23	17825	33718	2.47	1.31	0.56
High HDI								
2011		2.27	1.26	18974	36029	2.63	1.39	0.56
2012		2.32	1.28	19899	37917	2.76	1.45	0.55
2013		2.33	1.28	20524	39304	2.84	1.49	0.55
2014		2.33	1.26	20873	40344	2.91	1.50	0.54
2015		2.29	1.23	21039	40823	2.93	1.51	0.54
2016		2.25	1.20	21349	41443	2.95	1.52	0.53
2017		2.24	1.18	21565	42375	3.00	1.53	0.53
2018		2.25	1.17	22044	43790	3.09	1.56	0.52
2019		2.25	1.16	22642	45216	3.18	1.59	0.52
Low HDI	Male							
1990		1.68	1.23	4571	7055	1.16	0.75	0.73
1991		1.69	1.23	4692	7287	1.18	0.76	0.72
1992		1.68	1.22	4773	7431	1.19	0.76	0.72
1993		1.69	1.21	4891	7651	1.21	0.77	0.72
1994		1.69	1.21	5019	7861	1.23	0.78	0.72
1995		1.69	1.21	5128	8063	1.25	0.79	0.71
1996		1.69	1.20	5224	8285	1.27	0.80	0.71
Medium HDI								
1997		1.69	1.19	5321	8508	1.29	0.81	0.70
1998		1.71	1.19	5488	8831	1.33	0.83	0.70
1999		1.74	1.21	5724	9262	1.39	0.86	0.69
2000		1.82	1.25	6165	10041	1.50	0.92	0.69
2001		1.91	1.29	6598	10821	1.61	0.98	0.68
2002		2.01	1.35	7147	11816	1.74	1.06	0.67
2003		2.17	1.43	7871	13134	1.93	1.16	0.66
2004		2.34	1.53	8672	14629	2.14	1.27	0.65
2005		2.47	1.59	9325	15871	2.32	1.36	0.65
2006		2.56	1.63	9899	17039	2.48	1.44	0.64
2007		2.70	1.70	10618	18503	2.68	1.54	0.63
2008		2.89	1.80	11589	20386	2.94	1.67	0.62
2009		3.11	1.92	12673	22504	3.23	1.82	0.62
2010		3.35	2.03	13831	24833	3.56	1.98	0.61
High HDI								
2011		3.52	2.12	14896	26897	3.84	2.13	0.60
2012		3.64	2.18	15787	28654	4.07	2.24	0.60
2013		3.69	2.19	16342	29836	4.23	2.31	0.59
2014		3.67	2.15	16591	30576	4.31	2.34	0.59
2015		3.60	2.10	16679	30854	4.33	2.34	0.58
2016		3.53	2.06	16847	31167	4.35	2.35	0.58
2017		3.49	2.00	16901	31635	4.40	2.35	0.57
2018		3.48	1.97	17197	32532	4.50	2.38	0.57
2019		3.48	1.95	17608	33479	4.62	2.43	0.56
Low HDI	Female							
1990		1.17	0.69	2833	5335	0.93	0.49	0.59
1991		1.18	0.69	2908	5521	0.95	0.50	0.58
1992		1.17	0.68	2942	5603	0.96	0.50	0.58
1993		1.18	0.68	3007	5775	0.98	0.51	0.57
1994		1.17	0.66	3037	5887	0.98	0.51	0.57
1995		1.16	0.65	3065	6014	1.00	0.51	0.56
1996		1.16	0.64	3105	6175	1.01	0.51	0.55
Medium HDI								
1997		1.13	0.62	3097	6225	1.01	0.50	0.55
1998		1.12	0.61	3116	6338	1.02	0.50	0.54
1999		1.12	0.60	3192	6518	1.04	0.51	0.54
2000		1.12	0.60	3255	6643	1.05	0.52	0.54
2001		1.11	0.59	3299	6745	1.06	0.52	0.54
2002		1.10	0.59	3345	6834	1.07	0.52	0.53
2003		1.10	0.58	3419	7011	1.09	0.53	0.53
2004		1.11	0.58	3502	7255	1.12	0.54	0.52
2005		1.11	0.57	3556	7422	1.14	0.55	0.52
2006		1.11	0.56	3619	7639	1.17	0.55	0.51
2007		1.11	0.56	3683	7889	1.20	0.56	0.50
2008		1.12	0.55	3768	8167	1.24	0.57	0.49
2009		1.13	0.55	3876	8508	1.28	0.58	0.48
2010		1.15	0.55	3994	8885	1.33	0.60	0.48
High HDI								
2011		1.15	0.54	4078	9132	1.36	0.61	0.47
2012		1.13	0.52	4112	9263	1.38	0.61	0.47
2013		1.12	0.52	4181	9468	1.40	0.62	0.46
2014		1.12	0.51	4282	9768	1.44	0.63	0.45
2015		1.11	0.50	4360	9969	1.46	0.64	0.45
2016		1.11	0.50	4503	10275	1.50	0.66	0.45
2017		1.13	0.50	4664	10740	1.55	0.67	0.44
2018		1.15	0.50	4848	11258	1.62	0.70	0.44
2019		1.16	0.50	5034	11737	1.68	0.72	0.43

Times were categorised into four groups as per HDI value in 2019: very high (HDI>0.800), high (0.700 < HDI <0.799), medium (0.550 < HDI<0.699), and low (HDI<0.550). Data source: Global burden of disease 2019 study. Data source: MIR was calculated by the author using ASMR and ASIR data of oral cancer from the GBD 2019 study, and HDI data was procured from the UNDP database.

**Table 2:** Changes and trends of oral cancer at various stages of development in China.

Stages of development	Gender	Change in absolute number (%)		EAPC (95% CI)		
		Incident	Death	ASIR	ASMR	MIR
Low HDI (1990-1996)	Both sex	16.72	12.51	-0.05 (-0.23, 0.12)	-0.51 (-0.73, -0.29)	-0.44 (-0.69, -0.19)
Low HDI (1990-1996)	Male	17.43	14.29	3.75 (3.39, 4.11)	2.79 (2.48, 3.11)	-0.88 (-1.01, -0.76)
Low HDI (1990-1996)	Female	15.75	9.60	-0.40 (-0.79, -0.01)	-1.34 (-1.77, -0.92)	-0.92 (-1.08, -0.77)
Medium (1997-2010)	Both sex	128.86	111.75	0.08 (-0.03, 0.20)	-0.41 (-0.56, -0.26)	-0.40 (-0.62, -0.17)
Medium (1997-2010)	Male	191.99	159.93	5.64 (5.20, 6.08)	4.42 (4.01, 4.82)	-1.12 (-1.20, -1.04)
Medium (1997-2010)	Female	42.73	28.96	-0.55 (-1.13, 0.04)	-1.43 (-2.02, -0.83)	-0.86 (-1.00, -0.71)
High (2011-2019)	Both sex	25.50	19.33	-0.21 (-0.49, 0.06)	-1.33 (-1.75, -0.91)	-1.06 (-1.34, -0.78)
High (2011-2019)	Male	24.47	18.21	0.07 (-0.11, 0.24)	-0.95 (-1.04, -0.86)	-1.06 (-1.24, -0.87)
High (2011-2019)	Female	28.53	23.44	0.16 (-0.35, 0.67)	-0.87 (-1.30, -0.44)	-1.07 (-1.30, -0.83)

## Data Availability

The datasets generated and/or analysed during the current study are available in the GBD repository (http://ghdx.healthdata.org/gbd-results-tool) and the National Bureau of Statistics database of China (https://data.stats.gov.cn/index.htm).

## Abbreviations

OC: Oral cancer
HDI: Human development index
ASIR: Age-standardised incidence rates
ASMR: Age-standardised mortality rates
MIR: Mortality-to-incidence ratio
EAPC: Estimated annual percentage changes
CHE: Health expenditure as %age of GDP in calendar years
OOP: Out-of-pocket expenditure as %age of total health expenditure
NCD: Number of certified doctors per 10,000 population
HE: Per capita health expenditure
PM: Particulate matter.

## References

[1] Karunakaran K., Muniyan R. (2020). Genetic alterations and clinical dimensions of oral cancer: a review. *Molecular Biology Reports*.

[2] Torre L. A., Bray F., Siegel R. L., Ferlay J., Lortet-Tieulent J., Jemal A. (2015). Global cancer statistics, 2012. *CA: a Cancer Journal for Clinicians*.

[3] Ren Z. H., Xu J. L., Li B., Fan T. F., Ji T., Zhang C. P. (2015). Elective versus therapeutic neck dissection in node-negative oral cancer: evidence from five randomized controlled trials. *Oral Oncology*.

[4] Ren Z. H., Hu C. Y., He H. R., Li Y. J., Lyu J. (2020). Global and regional burdens of oral cancer from 1990 to 2017: results from the global burden of disease study. *Cancer Commun (Lond)*.

[5] Zhang L. W., Li J., Cong X. (2018). Incidence and mortality trends in oral and oropharyngeal cancers in China, 2005-2013. *Cancer Epidemiology*.

[6] International agency for research on cancer Global cancer observatory. https://gco.iarc.fr/today/online-analysis-table?v=2020&mode=cancer&mode_population=countries&population=900&populations=160&key=asr&sex=0&cancer=39&type=1&statistic=5&prevalence=0&population_group=0&ages_group%5B%5D=0&ages_group%5B%5D=17&group_cancer=1&include_nmsc=0&include_nmsc_other=1#collapse-by_country.

[7] Johnson N. (2001). Tobacco use and oral cancer: a global perspective. *Journal of Dental Education*.

[8] Sadri G., Mahjub H. (2007). Tobacco smoking and oral cancer: a meta-analysis. *J Res Health Sci*.

[9] Hu Y., Zhong R., Li H., Zou Y. (2020). Effects of betel quid, smoking and alcohol on oral cancer risk: a case-control study in Hunan Province, China. *Substance Use & Misuse*.

[10] Bezerra N. V., Leite K. L., de Medeiros M. M. (2018). Impact of the anatomical location, alcoholism and smoking on the prevalence of advanced oral cancer in Brazil. *Medicina Oral, Patología Oral y Cirugía Bucal*.

[11] Maxwell J. H., Grandis J. R., Ferris R. L. (2016). HPV-associated head and neck cancer: unique features of epidemiology and clinical management. *Annual Review of Medicine*.

[12] Wu C., Li M., Meng H. (2019). Analysis of status and countermeasures of cancer incidence and mortality in China. *Science China. Life Sciences*.

[13] Atun R., de Andrade L. O., Almeida G. (2015). Health-system reform and universal health coverage in Latin America. *Lancet*.

[14] Pakzad R., Mohammadian-Hafshejani A., Ghoncheh M., Pakzad I., Salehiniya H. (2015). The incidence and mortality of lung cancer and their relationship to development in Asia. *Transl Lung Cancer Res*.

[15] Harris J. A., Ritchie C. A., Hanna G. J., McCain J. P., Ji Y. D. (2021). The inequitable global burden of lip and oral cancers: widening disparities across countries. *Journal of Oral and Maxillofacial Surgery*.

[16] Hankey B. F., Ries L. A., Kosary C. L. (2000). Partitioning linear trends in age-adjusted rates. *Cancer Causes & Control*.

[17] Dong H., Duan S., Bogg L. (2016). The impact of expanded health system reform on governmental contributions and individual copayments in the new Chinese rural cooperative medical system. *The International Journal of Health Planning and Management*.

[18] Portes L. H., Machado C. V. (2015). WHO framework convention on tobacco control: adherence and establishment in Latin America. *Revista Panamericana de Salud Pública*.

[19] World Health Organization (WHO) (2018). *Global Status Report on Alcohol and Health 2018*.

[20] United Nation Development Programme Human development reports. http://www.undp.org/content/undp/en/home.html.

[21] Zhang X., Meng X., Chen Y., Leng S. X., Zhang H. (2017). The biology of aging and cancer: frailty, inflammation, and immunity. *Cancer Journal*.

[22] Zhou Z., Tang Q., Chen X., Yu T., Huang W., Liang F. (2021). The association between the socioeconomic status and systemic comorbidities in patients with oral cancers: a retrospective study in Guangxi Province. *Clinical Oral Investigations*.

[23] Cho H. J., Khang Y. H., Jun H. J., Kawachi I. (2008). Marital status and smoking in Korea: the influence of gender and age. *Social Science & Medicine*.

[24] Vega E., Reyes E., Ruiz H. (2004). Analysis of PM2.5 and PM10 in the atmosphere of Mexico City during 2000-2002. *Journal of the Air & Waste Management Association (1995)*.

[25] Chu Y. H., Kao S. W., Tantoh D. M., Ko P. C., Lan S. J., Liaw Y. P. (2019). Association between fine particulate matter and oral cancer among Taiwanese men. *Journal of Investigative Medicine*.

[26] Wang Y., Zhuang G., Tang A. (2005). The ion chemistry and the source of PM_2.5_ aerosol in Beijing. *Atmospheric Environment*.

[27] Kaur J., Sawhney M., DattaGupta S. (2013). Clinical significance of altered expression of *β*-catenin and E-cadherin in oral dysplasia and cancer: potential link with ALCAM expression. *PLoS One*.

[28] Qian X., Gu H., Wang L. (2018). Changes in smoking prevalence after the enforcement of smoking control regulations in urban Shanghai, China: findings from two cross-sectional surveys. *Tobacco Induced Diseases*.

[29] Zhu Y., Wen L. M., Li R., Dong W., Jia S. Y., Qi M. C. (2019). Recent advances of nano-drug delivery system in oral squamous cell carcinoma treatment. *European Review for Medical and Pharmacological Sciences*.

[30] World Health Organization Air quality in China. What can be done to improve air quality in China?. https://www.iqair.com/china.

[31] Omran A. R. (2001). The epidemiologic transition. A theory of the epidemiology of population change. 1971. *Bulletin of the World Health Organization*.

[32] Moi G. P., Silva A. M. C., Galvão N. D., de Castro M. M., Pereira A. C. (2018). Spatial analysis of the death associated factors due oral cancer in Brazil: an ecological study. *BMC Oral Health*.

[33] Chen D. T., Chou Y. F., Wu H. P. (2009). Income and the incidence of oral cavity cancer: cross-national study. *Journal of Otolaryngology - Head & Neck Surgery*.

[34] Hu Q. D., Zhang Q., Chen W., Bai X. L., Liang T. B. (2013). Human development index is associated with mortality-to-incidence ratios of gastrointestinal cancers. *World Journal of Gastroenterology*.

[35] Hu K., Lou L., Tian W., Pan T., Ye J., Zhang S. (2016). The outcome of breast cancer is associated with national human development index and health system attainment. *PLoS One*.

[36] Rafiemanesh H., Mehtarpour M., Khani F. (2016). Epidemiology, incidence and mortality of lung cancer and their relationship with the development index in the world. *Journal of Thoracic Disease*.

[37] Shao S. Y., Hu Q. D., Wang M. (2019). Impact of national human development index on liver cancer outcomes: transition from 2008 to 2018. *World Journal of Gastroenterology*.

[38] Sharma R. (2020). An examination of colorectal cancer burden by socioeconomic status: evidence from GLOBOCAN 2018. *The EPMA Journal*.

[39] Fitzmaurice C., Akinyemiju T. F., Al Lami F. H. (2018). Global, regional, and national cancer incidence, mortality, years of life lost, years lived with disability, and disability-adjusted life-years for 29 cancer groups, 1990 to 2016. *JAMA Oncology*.

[40] GBD 2016 Causes of Death Collaborators (2017). Global, regional, and national age-sex specific mortality for 264 causes of death, 1980-2016: a systematic analysis for the Global Burden of Disease Study 2016. *Lancet*.

